The article "A Mathematical Description of the Dynamics of Coronavirus Disease 2019 (COVID-19): A Case Study of Brazil" was published in 2020. Journal: Comput Math Methods Med.

# A Mathematical Description of the Dynamics of Coronavirus Disease 2019 (COVID-19): A Case Study of Brazil

**DOI:** 10.1155/2020/9017157

**Published:** 2020-09-30

**Authors:** Pedro V. Savi, Marcelo A. Savi, Beatriz Borges

**Affiliations:** Center for Nonlinear Mechanics, COPPE-Department of Mechanical Engineering, Universidade Federal do Rio de Janeiro, 21.941.972-Rio de Janeiro-RJ, Brazil P.O. Box 68.503

## Abstract

This paper deals with the mathematical modeling and numerical simulations related to the coronavirus dynamics. A description is developed based on the framework of the susceptible-exposed-infectious-removed model. Initially, a model verification is carried out calibrating system parameters with data from China, Italy, Iran, and Brazil. Results show the model capability to predict infectious evolution. Afterward, numerical simulations are performed in order to analyze different scenarios of COVID-19 in Brazil. Results show the importance of the governmental and individual actions to control the number and the period of the critical situations related to the pandemic.

## 1. Introduction

Coronavirus disease 2019 (COVID-19) is an illness that varies from a common cold to more severe diseases related to respiratory syndromes. It was discovered in 2019, being the first time the disease was identified in humans. It is related to the novel coronavirus (2019-nCoV), a zoonotic virus transmitted among animals and humans. On January 21, 2019, The World Health Organization (WHO) published the first Situation Report about the novel coronavirus that announces to the world the origin of the COVID-19, reporting cases of pneumonia of unknown etiology detected in Wuhan City, Hubei Province, China. Afterward, the situation evolves into a huge global crisis with severe effects in Italy, Iran, Spain, South Korea, and all over the world. On 11 March 2020, WHO declared COVID-19 as a pandemic.

This dramatic situation points out that all tools can be useful to plan the best strategies for the public health system. In this regard, mathematical modeling is an interesting approach that allows the evaluation of different scenarios, furnishing proper support for health system decisions. In general, the nonlinear dynamics of biological and biomedical systems is the objective of several research efforts that can be based on mathematical modeling or time series analysis [1]. In particular, coronavirus propagation can be described by a mathematical model that allows the nonlinear dynamics analysis, representing different populations related to the phenomenon.

The literature presents some examples related to the dynamics of infectious diseases. Different kinds of models can be employed, essentially considering nonlinear governing equations. Zhang et al. [2] investigated the cure effect on the virus model considering either cell-to-cell or cell-to-virus transmissions. Stability analysis is employed in order to evaluate the epidemiologic dynamical characteristics. Rihan et al. [3] described the dynamics of coronavirus infection in humans, establishing interaction among human cells and the virus.

Chen et al. [4] developed a mathematical model for calculating the transmissibility of the virus considering a simplified version of the bats-hosts-reservoir-people transmission model, defined as a reservoir-people model. Results follow the general trend of the initial propagation. Li et al. [5] estimated characteristics of the epidemiologic time distribution, exploiting some pattern trends of transmission propagation. Riou and Althaus [6] exploited the pattern of human-to-human transmission of a novel coronavirus in Wuhan, China. Two key parameters were considered: the basic reproduction number that defines the infectious propagation and the individual variation in the number of secondary cases. Uncertainty quantification tools were employed to define the transmission patterns.

Zou et al. [7] proposed a statistical model comparing the COVID-19 dynamics in several Asian countries, evaluating some of the essential populations related to the coronavirus disease. Another interesting approach for the COVID-19 modeling is presented by Car et al. [8] where a time series is employed to build a dataset for training a multilayer perceptron artificial neural network. This work concluded that the modeling of a disease using artificial intelligence could have a good agreement with real data.

Susceptible-exposed-infectious-removed (SEIR) models, and their variations, are an interesting approach to deal with the mathematical modeling of infectious diseases, being largely applied to describe HIV, Ebola, influenza, and Zika, among others. Pipatsart et al. [9] discussed infectious disease transmission on adaptive networks based on the susceptible-infectious-removed (SIR) model. Wu et al. [10] investigated coronavirus disease in the Wuhan-China case, evaluating nowcasting and forecasting domestic and international spread outbreak. Zeb et al. [11] investigated the SEIR model containing an isolated population that allows the description of isolation class. Lin et al. [12] proposed a model considering individual reaction, governmental action, and emigration. The model is based on the original work of He et al. [13] that proposed a model to describe the 1918 influenza. This model showed to be capable to capture the general propagation aspects of the novel coronavirus.

This paper proposes some adjustments in the original model due to Lin et al. [12] to describe COVID-19 dynamics. A different connection between infected and removed populations allows one to obtain a better match with real data. The proposed model is verified considering the infected population evolution of China, Italy, Iran, and Brazil. Afterward, Brazilian COVID-19 evolution is investigated, simulating different scenarios based on the governmental and individual reactions. The developed analysis considers average behaviors, neglecting spatial patterns. Results show that the model is able to capture the general behavior of the COVID-19 dynamics, being an important tool to guide decision-making.

## 2. Mathematical Model

A frame-by-frame description of the reality can be represented by a set of differential equations. By assuming only time evolution of state variables, *x* ∈ *ℜ*^*n*^, where spatial aspects are not of concern, it is possible to establish a governing equation of the form $\dot{x}=f\left(x\right),x\in {ℜ}^{n}$. The description of COVID-19 dynamics defines its propagation considering animal and human transmission. Different kinds of populations need to be defined in order to have a proper scenario of disease propagation.

Lin et al. [12] propose a susceptible-exposed-infectious-removed (SEIR) framework model to describe the COVID-19. This model was inspired by the original model of He et al. [13] for influenza. Essentially, the description considers a total population of size *N* that contains two classes: *D* is a public perception of risk regarding severe cases and deaths; and *C* represents the cumulative infected cases. In addition, the following populations are employed to describe the COVID-19 dynamics: *S* is the susceptible population, *E* is the exposed population, *I* is the infectious population, and *R* is the removed population that includes both recovered and deaths. A simplified version of the model considers only person-to-person transmission, and therefore, the zoonotic effect is neglected. This scenario assumes the second stage of the Wuhan-China case, after the close of the Huanan Seafood Wholesale Market. The emigration effect is also neglected in order to simplify the original model. Therefore, the governing equations consider the interaction among all these populations, being expressed by the following set of differential equations:

(1) $$\begin{array}{c} \dot{S}=-\beta \frac{SI}{N},\\ \dot{E}=\beta \frac{SI}{N}-\sigma E,\\ \dot{I}=\sigma E-\gamma I,\\ \dot{R}=\gamma_{R}I,\\ \dot{D}=d\gamma I-\lambda D,\\ \dot{C}=\sigma E, \end{array}$$

where the following parameters are defined: *γ* is the mean infectious period; *γ*_*R*_ is the adjusted removed period, defining the relation between the removed population and the infected one; *σ* is the mean latent period; *d* is the proportion of severe cases; and *λ* is the mean duration of public reaction. It should be pointed out that the parameter *γ* − *γ*_*R*_ defines the evolution of the nonreported removed population, which means that if *γ* = *γ*_*R*_, populations are restricted to the classical SEIR case.

The function *β* = *β*(*t*) represents the transmission rate that considers governmental action, represented by (1 − *α*), and the individual action, represented by the function (1 − (*D*/*N*))^*κ*^. Therefore, the transmission rate is modeled as follows:

(2) $$\begin{array}{c} \beta =\beta \left(t\right)={\hat{\beta }}_{0}\left(1-\hat{\alpha }\right)\delta , \end{array}$$

where ${\hat{\beta }}_{0}=\beta_{0}^{\left(i\right)}H\left(t-T_{\beta_{0}}^{\left(i\right)}\right)$ represents the nominal transmission rate and *H*(*t* − *T*_*β*_0__^(*i*)^) is a step function with the form illustrated in Figure 1. Its use is convenient in order to contemplate variations of the transmission rate through time, being defined as follows.

(3) $$\begin{array}{c} H\left(t-T_{\beta_{0}}^{\left(i\right)}\right)=\left\{\begin{array}{c} \beta_{0}^{\left(1\right)},\;\text{if }t\leq T_{\beta_{0}}^{\left(1\right)},\\ \beta_{0}^{\left(2\right)},\;\text{if }t\leq T_{\beta_{0}}^{\left(2\right)},\\ \beta_{0}^{\left(3\right)},\;\text{if }t\leq T_{\beta_{0}}^{\left(3\right)},\\ \vdots \end{array}\right. \end{array}$$

This general function can represent constant values or different step functions. Using the same strategy, the governmental action is described as follows:

(4) $$\begin{array}{c} \hat{\alpha }=\alpha_{i}\;H\left(t-T_{\text{Gov}}^{\left(i\right)}\right), \end{array}$$

where different steps are considered defined by time instants *T*_Gov_^(*i*)^.

Individual action is represented by the following equation:

(5) $$\begin{array}{c} \delta ={\left(1-\frac{D}{N}\right)}^{\kappa }, \end{array}$$

where the intensity of responses is defined by parameter *κ*. These parameters need to be adjusted for each place, being essential for the COVID-19 description.

In general, parameter definitions depend on several issues, being a difficult task to be adjusted. In this regard, it should be pointed out that real data has spatial aspects that are not treated by this set of governing equations. Hence, this analysis is a kind of average behavior that needs a proper adjustment to match real data. Besides, Li et al. [14] evaluated the Wuhan situation concluding that undocumented novel coronavirus infections are critical for understanding the overall prevalence and pandemic potential of this disease. The authors estimated that 86% of all infections were undocumented and that the transmission rate per person of undocumented infections was 55% of documented infections. This aspect makes the description even more complex.

The use of step functions to define some parameters introduces a time-dependent description, allowing a proper representation of different scenarios. This is especially important for the representation of the transmission rate. It is also important to observe that either governmental or individual actions have a delayed effect on system dynamics that can be adjusted by this time-dependent behavior. Virus mutations are another relevant aspect related to the description of COVID-19 dynamics that can dramatically alter the system response but are not treated here.

Numerical simulations are carried out considering the fourth-order Runge-Kutta method. The next sections treat the COVID-19 dynamics considering two different objectives. Initially, the next section performed a model verification using information from China, Italy, Iran, and Brazil. Afterward, the subsequent section evaluates different scenarios for the Brazilian case, using the parameters adjusted on the verification cases.

## 3. Model Verification

As an initial step of the COVID-19 dynamical analysis, a model verification is carried out using information available on Worldometer (https://www.worldometers.info/coronavirus/), considering information from China, Italy, Iran, and Brazil (last updates: China, March 26; Italy, March 21; Iran, March 26; and Brazil, March 24). The fundamental hypothesis of the analysis is that the average population of the country is of concern. Therefore, it is assumed that each country has a homogeneous distribution, without spatial patterns.

Different country information is useful to calibrate the model parameters, evaluating its correspondence with real data.  Table 1 presents the parameters employed for all simulations. They are based on the information of Lin et al. [12] that, in turn, is based on other references such as He et al. [15] and Breto et al. [16]. For more details, see other citations referenced therein.

Susceptible population initial condition is assumed to be *S*_0_ = 0.9*N* − *E*_0_ − *I*_0_ − *R*_0_. In addition, it is adopted that, initially, there is no removed population, i.e., *R*_0_ = 0. Another information needed for the model is the number of exposed persons for each infected person. It is assumed that each infected person has the potential to expose 20 persons, *E*_0_ = 20*I*_0_.

The transmission rate considers specific parameters for each case. Nevertheless, the reference values are presented in Table 2.

Other parameters are adjusted depending on the treated case. In the sequence, the dynamics of four different countries is analyzed in order to promote a model verification.

### 3.1. Verification Simulations

The first scenario for the model verification is based on China results. It should be pointed out that this analysis considers all cases in China, not restricted to Wuhan. Due to chronological issues, the Chinese case is the one with a large number of real data, which makes it useful to describe the whole process. Parameters presented in Table 3 are employed for simulations with a population of *N* = 1.43 × 10^9^ and an initial state with 554 infected persons (*I*_0_ = 554). It should be highlighted again that these parameters are average ones, representing a whole country average, adjusted in a phenomenological way. Of course, reaction time is different from the distinct parts of the country, which makes it necessary to estimate parameters based on the real data in an average way.  Figure 2 presents the infected population evolution showing a good agreement between the simulation and real data. A comparison of the model prediction error compared with real data is interesting to verify the model capability to describe the COVID-19 dynamics.  Figure 3 presents daily errors from China, highlighting the average and maximum errors. Note that the maximum error is less than 28%, with an average error of 13.58%.

For the following three cases, Italy, Iran, and Brazil, it is assumed that the second stage of governmental action has not been reached yet. Therefore, it is represented by a step function *α*_*i*_ = [0, 0.4239], which means that *T*_Gov_^(2)^ is neglected and *α*_3_ does not exist.

The Italian case is now in focus considering parameters presented in Table 4 with a population of *N* = 60.48 × 10^6^ and an initial state with 20 infected persons (*I*_0_ = 20). A step function is considered to define the nominal transmission rate, *β*_0_, due to extreme governmental actions that have not been effective until the present days.  Figure 4 presents the infected population simulation compared with real data, showing a good agreement.  Figure 5 presents daily errors from Italy, highlighting the average and maximum errors. In this case, the maximum error is less than 19%, with an average error of 10.60%.

The Iran case is evaluated assuming parameters presented in Table 5 with a population of *N* = 81.16 × 10^6^ and an initial state with 20 infected persons (*I*_0_ = 20). Results are presented in Figure 6 showing a good agreement with real data.  Figure 7 presents daily errors, highlighting the average and maximum errors. Although the average error is 15.46%, the maximum error is around 42%, which is a large value. Nevertheless, it should be observed that the big values are related to the beginning of the predictions, probably due to the characteristics of the reported real data.

The Brazilian case is now of concern considering parameters presented in Table 6 with a population of *N* = 209.3 × 10^6^ and an initial state with 10 infected person (*I*_0_ = 10).  Figure 8 presents the infected population evolution showing that the same trend of the other cases is followed, being enough to have a general scenario. It should be highlighted that the Brazilian outbreak is in the beginning, with information that is not enough for better calibration.

## 4. Brazilian Scenarios

This section has the objective to investigate different scenarios related to COVID-19 dynamics in Brazil. Parameters adjusted in the previous section are employed to evaluate different scenarios varying the governmental and individual reactions. It should be pointed out that this adjustment does not have enough information, but it is possible to perform at least a qualitative analysis of the COVID-19 dynamics in Brazil.

Initially, two different transmission rates are defined: without intervention (*α* = *κ* = 0), naive scenario, and with the governmental and individual actions (*α* ≠ 0; *κ* ≠ 0).  Figure 9 presents numerical simulations together with the real data that is presented just for the first days. The same parameters presented in Table 6 are employed assuming *T*_Gov_^(2)^ = 37 days. A logarithm scale is adopted since the naive scenario has a dramatic increase in infected cases. Besides the big difference between both cases, it is clear the huge impact of variations on the transmission rate function that represents the governmental and individual actions. It is noticeable that effective actions tend to reduce the infected population, reducing the final crisis period as well.

A more detailed analysis of the COVID-19 dynamics is treated considering the other populations for the case with intervention treated in Figure 9 (parameters of Table 6 with *T*_Gov_^(2)^ = 37 days).  Figure 10 presents all system state variables, showing the susceptible, *S*, exposed, *E*, infected, *I*, removed, *R*, public perception, *D*, and cumulative cases, *C*. The interaction among all the populations defines a kind of equilibrium established by the governing equations.

Nowadays, one of the most relevant issues to be discussed in terms of propagation is the governmental and individual actions. A parametric analysis is of concern considering distinct scenarios related to intervention. Scenarios defined by the variation of the intervention moments are initially treated. The moment of the governmental action start, represented by the parameter *T*_Gov_^(1)^ (day), is analyzed in Figure 11, considering the following values: 17, 22, 27, and 32, and *T*_Gov_^(2)^ is assumed to be 20 days after *T*_Gov_^(1)^. Note that the delay to the start of the governmental action dramatically alters the response, increasing the number of infected populations and its duration. The same conclusion can be established considering the second governmental action, represented by *T*_Gov_^(2)^ (day), presented in Figure 12 that shows the same trend considering a different set of start instants: 37, 42, 47, and 52.

A scenario with a governmental action that starts, finishes, and then restarts again is now evaluated, considering the following parameters: *T*_Gov_^(*i*)^ = [17, 37, 52] and *α*_*i*_ = [0, 0.4239, 0, 0.8478]. This scenario is compared with the usual one where the intervention starts at a level and then evolves to a more severe situation, considering *T*_Gov_^(*i*)^ = [17, 52] and *α*_*i*_ = [0, 0.4239, 0.8478].  Figure 13 shows both situations represented by the transmission function and the evolution of infected populations. It is clear that the interruption of the governmental action causes a dramatic worst scenario.

## 5. Conclusions

A mathematical model based on the susceptible-exposed-infectious-removed framework is employed to describe the COVID-19 dynamics. A verification procedure is performed based on the available data from China, Italy, Iran, and Brazil. Afterward, different scenarios from Brazil are analyzed. Results clearly show that the governmental and individual actions are essential to reduce the infected populations and also the total period of the crisis. In this regard, it is observed that the infected peak reduction is usually associated with a smaller period of the critical infected population. In addition, another important conclusion is that the precipitate finish of social isolation can have a dramatic influence on virus propagation, increasing significantly the infected population. The mathematical model can be improved in order to include more phenomenological information that can increase its capability to describe different scenarios. Nevertheless, it should be pointed out that mathematical modeling and numerical simulations are important tools that can be essentially useful for public health planning.

## Figures and Tables

**Figure 1:** Step function employed to consider parameter variations through time.

**Figure 2:** China: infected population through time.

**Figure 3:** China: prediction errors between the simulated and real data of the infected population.

**Figure 4:** Italy: infected population through time.

**Figure 5:** Italy: prediction errors between the simulated and real data of the infected population.

**Figure 6:** Iran: infected population through time.

**Figure 7:** Iran: prediction errors between the simulated and real data of the infected population.

**Figure 8:** Brazil: infected population through time.

**Figure 9:** Transmission evolution considering two different scenarios for different transmission rates: without intervention (*α* = *κ* = 0), naive scenario, and with governmental intervention and individual action with the values adjusted in the previous section.

**Figure 10:** Population interactions considering a scenario with intervention: susceptible, *S*, exposed, *E*, infected, *I*, removed, *R*, public perception, *D*, and cumulative cases, *C*.

**Figure 11:** Infected population evolution considering the different first governmental action start, represented by the parameter *T*_Gov_^(1)^ (day): 17, 22, 27, and 32.

**Figure 12:** Infected population evolution considering the different second governmental action start, represented by the parameter *T*_Gov_^(2)^ (day): 37, 42, 47, and 52.

**Figure 13:** Infected population evolution considering different scenarios related to the governmental action, $\hat{\alpha }$.

**Table 1:** Model parameters.

Parameter	Description	Value
*σ* ^−1^	Mean latent period	3 days
*γ* ^−1^	Mean infectious period	5 days
*γ*_*R*_^−1^	Adjusted removed period	22 days
*d*	Proportion of severe cases	0.2
*λ* ^−1^	Mean duration of public reaction	11.2 days

**Table 2:** Reference parameters for the transmission rate.

Parameter	Value
*α*_*i*_	[0, 0.4239, 0.8478]
*κ*	1117.3

**Table 3:** Model parameters for the transmission rate of China.

Parameter	Value
*β*_0_	0.514
*T*_Gov_^(*i*)^	[13, 29] days

**Table 4:** Model parameters for the transmission rate of Italy.

Parameter	Value
*β*_0_^(*i*)^	[0.594, 1.1]
*T*_*β*_0__^(1)^	22 days
*T*_Gov_^(1)^	22 days

**Table 5:** Model parameters for the transmission rate of Iran.

Parameter	Value
*β*_0_^(1)^	0.594
*T*_Gov_^(1)^	24 days

**Table 6:** Model parameters for the transmission rate of Brazil.

Parameter	Value
*β*_0_^(1)^	0.675
*T*_Gov_^(1)^	17 days

## Data Availability

The data used to support the findings of this study are included within the article.
